# Association of Obstructive Sleep Apnea Syndrome (OSA/OSAHS) with Coronary Atherosclerosis Risk: Systematic Review and Meta-Analysis

This article has been retracted.

**DOI:** 10.1155/2022/8905736

**Published:** 2022-08-17

**Authors:** Liwen Chen, Shujing Zou, Jinhong Wang

**Affiliations:** Department of Respiration, The Third Affiliated Hospital, Southern Medical University, Guangzhou, China 510630

## Abstract

**Objective:**

Obstructive sleep apnea syndrome (OSA) is the most common type of sleep disorders. This study aimed to systematically review the correlation between OSA and the risk of coronary atherosclerosis.

**Methods:**

Literature on case-control studies on the relationship between coronary heart disease (CHD) and sleep apnea syndrome was collected and collated, and the incidence of SAS in CHD and non-CHD patients was observed and compared. RevMan 5.2 analysis software and Stata12SE analysis software were used for heterogeneity test and combination analysis of the included studies. The results were expressed with odds ratio (OR), 95% confidence intervals (CI) were calculated, and publication bias and sensitivity tests were evaluated.

**Results:**

There was a statistical difference in OSA associated with the risk of coronary atherosclerosis between the experimental group and the control group [OR = 1.38, 95% CI (1.18, 1.62), *P* < 0.0001, *I*^2^ = 0%, *Z* = 3.93]. OSA associated with vascular endothelial injury [OR = 3.59, 95% CI (3.00, 4.29), *P* < 0.00001, *I*^2^ = 90%, *Z* = 14.09]. OSA is associated with vascular oxidation emergency [OR = 2.19, 95% CI (2.05, 2.33), *P* < 0.00001, *I*^2^ = 94%, *Z* = 23.40]; OSA is associated with chronic vascular inflammation [OR = 1.70, 95% CI (1.39, 2.07), *P* < 0.00001, *I*^2^ = 16%, *Z* = 5.18].

**Conclusion:**

The incidence of obstructive sleep apnea in patients with CHD was higher than that in non-CHD patients, and obstructive sleep apnea was a risk factor for CHD.

## 1. Introduction

Coronary heart disease is closely related to OSA/OSAHS [1]. At present, there are already at home and abroad, and there are many case-control studies on the relationship between coronary heart disease and SAS, but they are generally limited to small sample size and large selection bias [2–4]. Obstructive sleep apnea syndrome (OSAS) is airway obstruction that can lead to significant physiologic disturbance with numerous clinical impacts. Sleep apnea syndrome (SAS) is a potentially dangerous disease with high morbidity. According to the etiology, it can be divided into obstructive, central, mixed, and obstructive sleep apnea syndrome. OSAS is the most common. Multiple regression analysis has confirmed that SAS is a risk factor for unstable angina pectoris and myocardial infarction, but there is still a lack of large-scale clinical studies in China [5]. The occurrence of OSA is as high as 40% to 80% in patients with hypertension, coronary artery disease, heart failure, and pulmonary hypertension. Despite its high prevalence in patients with heart disease patients, OSA is often underrecognized and undertreated in cardiovascular practice.

The introduction of the 2021 American Heart Association/American Foundation of Cardiology Scientific Statement on Sleep apnea and Cardiovascular Disease has led to recognition of the impact of sleep apnea on cardiovascular disease. Early detection and timely correction of sleep apnea play an important role in the secondary prevention of coronary heart disease (coronary heart disease). Foreign epidemiological data show that SAS is a disease with high morbidity and high risk [6]. The incidence of adult sleep apnea is 4%~7%, and OSAS accounts for more than 90%, adult male 4% and female 2%. The incidence increases with the increase of age, and the incidence of the elderly over 50 years old >6%. According to the preliminary epidemiological survey of OSAS in China, the prevalence rate is about 4% [7]. Based on the population of 1.3 billion in China, there are at least 52 million OSAS patients [8].

An increase in baseline BMI of kg/m^2^ was associated with a 12% increased risk of coronary heart disease. Body mass index was closely correlated with apnea/hypopnea index, respiratory disorder index and oxygen saturation index, and independently correlated with apnea/hypopnea index. Apnea hypopnea index was also an independent risk predictor of CHD death in a follow-up study [9]. The possible mechanism of sleep disorders in obese patients is as follows: the increase of body mass in obese patients affects the thorax and abdomen, reduces the compliance of chest wall, reduces the volume of lung tissue, and aggravates the mechanical load of respiratory system. As a result, the functional residual volume decreases, especially in the supine position. Obesity causes sleep apnea mainly by increasing the soft tissue around the upper respiratory tract, changing the structure of nonrespiratory tract, resulting in respiratory tract stenosis [10]. And because the adipose tissue around the respiratory tract increases, the muscular tissue decreases, and the fibrous connective tissue increases, and the upper respiratory tract becomes relaxed. When inhaled, the upper respiratory tract collapsed, increasing the mechanical load of respiration. On the basis of narrow upper respiratory tract, the damage of respiratory function was further aggravated. SAS is based on the repeated occurrence of upper respiratory tract obstruction, resulting in apnea and insufficient ventilation, repeated awakening, and so on, resulting in repeated hypoxemia, hypercapnia, and acidic environment in the body. More patients with sleep apnea combined with coronary heart disease developed angina pectoris at night, suggesting an imbalance between myocardial oxygen supply and myocardial oxygen consumption, which may play a role through the following mechanisms.

In this study, meta-analysis was conducted on domestic and foreign clinical case-control studies on the relationship between coronary heart disease and OSA to obtain comprehensive quantitative analysis results of the relationship between coronary heart disease and OSA, so as to make up for the deficiency of single studies and provide more reliable evidence-based medical evidence.

## 2. Materials and Methods

### 2.1. Literature Retrieval Strategy

The main retrieval words were “coronary heart disease, sleep apnea syndrome, coronary artery disease, CAD, Sleep apnea syndrome, obstructive sleep apnea syndrome.” Combined with CAD and CHD, SAS and OSAHS ensure the comprehensiveness of the index. China National Knowledge Infrastructure (CNKI), CBMdisc, VIP, Wanfang, PubMed, Embase, Cochrane, and Google Scholar were searched by computer, supplemented by literature retrospective and manual retrieval methods. All literatures on the relationship between coronary heart disease and obstructive sleep apnea syndrome were retrieved from the self-established database up to December 31, 2021 (Figure 1).

### 2.2. Literature Inclusion Criteria

The literature inclusion criteria were as follows: ① open and unpublished primary literature; ② the original data are complete; and ③ patients with coronary heart disease and noncoronary heart disease. The incidence of OSA was a case-control study. ④ The diagnostic criteria of coronary heart disease are the same. According to the American College of Cardiology (ACC) and the American Heart Association (AHA) coronary angiography (CAG) guidelines, CAG demonstrates ≥50% stenosis of 1 or more coronary vessels. The diagnostic criteria for OSA are the same. Apnea was defined by polysomnogram (PSG) as at least 10 s of airflow cessation from the nose and mouth. Hypopnea was defined as a 50% reduction in airflow, lasting more than 10 s, with a corresponding decrease in oxygen saturation of ≥4%. OSA was diagnosed with sleep apnea hypopnea index (AHI) ≥5 or PSG for more than 30 recurrent episodes of apnea and hypopnea during 7 hours of sleep per night. Because some studies used AHI≥10 as SAS diagnostic criteria, we analyzed the differences according to the diagnostic criteria.

### 2.3. Literature Exclusion Criteria

The literature exclusion criteria are as follows: ① review literature and other nonprimary literature; ② there is no literature for extracting data; ③ studies without clear definition of diagnostic criteria for coronary heart disease and obstructive sleep apnea syndrome; and ④repeated publication of literature.

### 2.4. Literature Quality Evaluation

The selected studies were case-control studies. The Newcastle-Ottawa Scale (NOS) was used to score literature quality, and independent evaluations were carried out in pairs in terms of case selection and group control conditions, intergroup comparability, and similarity of exposure factors. Differences were discussed and resolved. If the problem is still unresolved, it will be submitted to the third party for evaluation. The full score was 9 stars, and literatures with a total score of more than 5 stars could be included in the meta-analysis (Figure 2).

### 2.5. Heterogeneity Test and Meta-Analysis

If the evaluation results showed no publication bias, the heterogeneity test was carried out among the studies. If there was no heterogeneity among the studies, the fixed-effect model was used for analysis. If heterogeneity exists between studies, random effects model is used to analyze. Meta-analysis was performed using RevMan 5.2 software. The results were expressed with odds ratio (OR), and the 95% confidence interval (95% CI) was calculated. When OR = 1, OR 95% CI including 1, *P* > 0.05, that is, the difference is not statistically significant. When the upper and lower bounds of 95% CI did not contain 1, *P* < 0.05, the difference was statistically significant (Figure 3).

Population (P): Patients meets the diagnostic criteria of coronary heart disease

Intervention (I): Whether patients had OSA

Comparison (C): The control was whether patients in these diseases were diagnosed with OSA

Outcome measures (O): OSA associated with the risk of coronary atherosclerosis, vascular endothelial injury, vascular oxidation emergency, and chronic vascular inflammation

Study design (S): Retrospective analysis

### 2.6. Sensitivity Analysis

Stability sensitization of the results was observed by eliminating important studies that might influence the analysis and by transforming the effect model perceptual analysis.

### 2.7. Statistical Analysis

All statistical calculations were carried out using SPSS statistical software. Because Stata analysis software can provide quantitative analysis of publication bias, Sata12 software is used for publication bias evaluation. If there is publication bias, the method of “Cutting and filling” is used to correct it. If it cannot be corrected, discussion of publication bias can only be conducted. *P* values <0.05 were considered significant.

## 3. Result

### 3.1. Results of Literature Quality Evaluation

A total of 351 literatures related to coronary heart disease and obstructive sleep apnea syndrome were retrieved, including 14 literatures [11–24] after independent screening and evaluation by two persons. Although 9 of the excluded literatures were case-control studies of coronary heart disease, coronary angiography was not performed in 6 of the excluded literatures, and the diagnostic criteria of obstructive sleep apnea syndrome were not clearly indicated in 3 of the excluded literatures. 9 control studies used AN AHI≥5 as a diagnostic criterion for OSA, and five control studies used an AHI≥10 as a diagnostic criterion for OSA (Table 1).

### 3.2. OSA Associated with the Risk of Coronary Atherosclerosis

Among the 14 RCTs literatures included in OSA associated with the risk of coronary atherosclerosis, heterogeneity test was carried oysis for 4 included literatures, so there was a statistical difference in OSA associated with the risk of coronary atherosclerosis between the experimental group and the control group [OR = 1.38, 95% CI (1.18, 1.62), *P* < 0.0001, *I*^2^ = 0%, *Z* = 3.93] (Figure 4).

### 3.3. OSA Associated with Vascular Endothelial Injury

Among the 14 RCTs literatures included in OSA associated with vascular endothelial injury, heterogeneity test was carried oysis for 4 included literatures, so there was a statistical difference in OSA associated with vascular endothelial injury between the experimental group and the control group [OR = 3.59, 95% CI (3.00, 4.29), *P* < 0.00001, *I*^2^ = 90%, *Z* = 14.09] (Figure 5).

### 3.4. OSA Associated with Vascular Oxidation Emergency

Among the 14 RCTs literatures included in OSA associated with vascular oxidation emergency, heterogeneity test was carried oysis for 4 included literatures, so there was a statistical difference in OSA associated with vascular oxidation emergency between the experimental group and the control group [OR = 2.19, 95% CI (2.05, 2.33), *P* < 0.00001, *I*^2^ = 94%, *Z* = 23.40] (Figure 6).

### 3.5. OSA Associated with Chronic Vascular Inflammation

Among the 14 RCTs literatures included in OSA associated with chronic vascular inflammation, heterogeneity test was carried oysis for 4 included literatures, so there was a statistical difference in OSA associated with chronic vascular inflammation between the experimental group and the control group [OR = 1.70, 95% CI (1.39, 2.07), *P* < 0.00001, *I*^2^ = 16%, *Z* = 5.18] (Figure 7).

## 4. Discussion

The selected studies in this study were verified to have no publication bias, and sensitivity analysis also showed that the results of this study were relatively stable [25]. Therefore, it can be considered that the effect of this study is relatively reliable. Among all 14 studies included in this study, the 95% CI of 2 included 1, indicating that the difference was not statistically significant and could not indicate that OSA was a risk factor for coronary heart disease [26]. The OR value of 12 studies was greater than 1, and the 95% CI lower limit was greater than 1, indicating that OSA is a risk factor for coronary heart disease [27]. However, after the integration and analysis of individual studies, the OR values were all greater than 1, and the 95% CI lower limit was greater than 1, and the *P* values were all less than 0. 05, indicating statistically significant differences [28–31]. These results indicated that after multiple studies were combined, OSA was still positively associated with the occurrence of coronary heart disease, and OSA was a risk factor for coronary heart disease [32]. Moreover, the 95% CI interval after economic cooperation and integration is significantly reduced, which makes the reliability of the sample index to estimate the overall parameters better.

Conclusion based on single research results is difficult to reflect the essence of things and may result in accidental results due to the action of a variety of factors [33]. Meta-analysis is a research method that systematically analyzes and quantitatively synthesizes the results of multiple independent studies with the same research purpose [34]. The purpose is to improve the statistical test efficiency, evaluate the inconsistencies or contradictions of research results, find the shortcomings of a single study, and process a large number of literatures, which is not limited by the number of studies [35–37]. It plays an important role in clinical diagnosis, treatment, risk assessment, preventive intervention, health service, and decision-making. Due to the small sample size of clinical case studies of OSA and CHD, this paper provides a quantitative average effect or correlation combined with multiple studies, which makes the confidence interval more convergent. The results of each study are more comprehensive and quantitative, and the conclusion is more comprehensive and reliable. OSA contributes to the occurrence of CHD through a variety of mechanisms, but the specific mechanisms have not been fully elucidated. OSA induced apnea, and chronic intermittent hypoxia and sleep structure disorders can cause a series of pathophysiological changes such as hemodynamic changes, sympathetic nervous activity increases, and vascular endothelial dysfunction, which are conducive to the occurrence of coronary heart disease [38]. The main pathological mechanism of coronary heart disease : pathophysiological changes, such as increased left ventricular load, sympathetic-parasympathetic imbalance, oxidative stress, inflammation and vascular endothelial dysfunction, promote and aggravate the occurrence and development of coronary atherosclerosis, and ultimately lead to coronary heart disease [39].

The advantage of this study was to analyze the incidence of obstructive sleep apnea in patients with CHD, which will provide solid foundation for future treatment. However, there are also shortcomings of this study: (1) In addition to OSA as the main observational factor in the included study, there are many other coronary heart disease risk factors, and it is difficult to use meta-analysis to combine correction or exclude the influence of other treatment factors; (2) meta-analysis is not an experimental study, and there may be a variety of bias; and (3) all included studies were hospital-based case-control studies. According to the NOS scale, it is impossible to evaluate the quality of all literature.

## 5. Conclusion

The incidence of obstructive sleep apnea in patients with CHD was higher than that in non-CHD patients, and obstructive sleep apnea was a risk factor for CHD.

## Figures and Tables

**Figure 1:** Flow chart of the literature screening.

**Figure 2:** Literature quality evaluation chart. (a) Risk of bias graph. (b) Risk of bias summary.

**Figure 3:** (a–d) Funnel plot of literature publication bias.

**Figure 4:** Meta-analysis of OSA associated with the risk of coronary atherosclerosis between two groups.

**Figure 5:** Meta-analysis of OSA associated with vascular endothelial injury between two groups.

**Figure 6:** Meta-analysis of OSA associated with vascular oxidation emergency between two groups.

**Figure 7:** Meta-analysis of OSA associated with chronic vascular inflammation between two groups.

**Table 1:** Basic clinical features of 14 literatures were included in our study.

Study	Age	Gender(man)	Experimental group(*N*)	Control group(*N*)	NOS score	Research type
Ogilvie RP 2018 [11]	43.71 ± 2.2	41.25%	2210/3874	1664/3874	8	RCT
McEvoy RD 2016 [12]	55.65 ± 3.4	69.12%	1700/2717	1017/2717	7	RCT
Zinchuk AV 2021 [13]	53.12 ± 4.5	45.72%	149/249	100/249	8	RCT
Celik Y 2021 [14]	42.15 ± 4.5	44.12%	108/208	100/208	8	RCT
Glantz H 2013 [15]	52.85 ± 1.4	51.89%	362/662	300/662	8	RCT
Glantz H 2015 [16]	54.36 ± 1.2	63.45%	311/431	120/431	7	RCT
Balcan B 2019 [17]	62.62 ± 2.2	78.10%	69/99	72/104	9	RCT
Thunström E 2017 [18]	42.61 ± 3.0	48.75%	119/220	101/220	9	RCT
Liu X 2014 [19]	57.25 ± 4.5	59.23%	32/40	26/40	7	RCT
Balcan B 2020 [20]	48.22 ± 5.2	56.22%	135/244	109/244	8	RCT
Lewis EF 2017 [21]	51.35 ± 1.1	53.16%	200/318	118/318	8	RCT
Huang Z 2016 [22]	61.25 ± 1.0	66.34%	40/70	30/70	8	RCT
Glantz H 2017 [23]	51.45 ± 1.2	68.25%	145/244	95/244	7	RCT
Sánchez-de-la-Torre A 2016 [24]	64.22 ± 1.1	56.68%	499/796	297/796	7	RCT

## Data Availability

The data used to support this study is available from the corresponding author upon request.
